# An Artificial Neural Network Algorithm for the Evaluation of Postoperative Rehabilitation of Patients

**DOI:** 10.1155/2021/3959844

**Published:** 2021-10-11

**Authors:** Kunhao Tang, Ruogu Luo, Sanhua Zhang

**Affiliations:** Department of Computer and Engineering, Hunan Institute of Technology, HengYang 421002, China

## Abstract

In order to explore the application of artificial neural network in rehabilitation evaluation, a kind of ANN stable and reliable artificial intelligence algorithm is proposed. By learning the existing clinical gait data, this method extracted the gait characteristic parameters of patients with different ages, disease types and course of disease, and repeated data iteration and finally simulated the corresponding gait parameters of patients. Experiments showed that the trained ANN had the same score as the human for most of the data (82.2%, Cohen's kappa = 0.743). There was a strong correlation between ANN and improved Ashworth scores as assessed by human raters (*r* = 0.825, *P* < 0.01). As a stable and reliable artificial intelligence algorithm, ANN can provide new ideas and methods for clinical rehabilitation evaluation.

## 1. Introduction

Artificial intelligence (AI) has become a neighborhood with many practical applications and active research topics. Artificial neural network (ANN), as an important branch of modern artificial intelligence technology, has been widely and deeply applied to modern medical activities due to its powerful learning ability and stable feature recognition and prediction functions [1]. Rehabilitation assessment is mainly a quantitative or qualitative description of patients' functional status, including physical motor function assessment, balance assessment, and other dimensions. However, at present, many rehabilitation assessment methods are time-consuming and laborious and difficult to accurately quantify [2]. Therefore, in recent years, artificial intelligence experts have designed and developed a variety of ANN algorithms, and in the real clinical environment to evaluate the rehabilitation of patients, they have achieved satisfactory results. As an artificial intelligence tool, the artificial neural network has been widely used in the clinical diagnosis of diseases such as tumor and pulmonary embolism since the 1990s. Dr. Robert H. Nielsen, the inventor of the neural computer, defined the neural network as a computing system composed of many simple and highly interconnected processing elements, which can deal with real problems by dynamically reacting to external input information [3]. Stroke has become a common disease in clinical practice due to its high morbidity and disability rate. It is often accompanied by a variety of functional disorders, among which the upper limb motor dysfunction is the most widely affecting limb dysfunction. Recently, rehabilitation medicine is gradually developing towards the direction of precision, long-distance, intelligence, and individuation, among which precise evaluation is an important direction. Based on the fusion of sensor technology and artificial intelligence theory, the automatic evaluation of upper limb motor function is deeply studied, and the motion measurement system is designed from the motor dysfunction of arm, hand, and upper limb activity function. Three different depth learning methods based on sensor data are proposed to realize the feature extraction of clinical scale [4].

Pryor et al. proposed a body evaluation model based on the mixed density neural network. The movement sequences of patients were collected by the Microsoft Kinect sensor as the input of the neural network. The neural network consists of two layers: self-coding layer and mixed density layer. The former is used to reduce the dimension of the motion sequence and extract the features, while the latter is used to express the patient's motion sequence as a Gaussian density function and compare it with the preset motion to evaluate the patient's body function. This model can be applied to the rehabilitation evaluation and training guidance of stroke rehabilitation patients in the family environment [5]. Wilkinson et al. used clustering analysis and artificial neural network to analyze the gait data of 74 stroke patients obtained by the three-dimensional motion analysis system. First, they performed clustering analysis on the gait patterns of patients through K-means algorithm, the characteristics used included 14 parameters such as the landing position of the patient's foot, and three patient clusters were obtained. The first touching position of the foot was found to correspond to the forefoot, foot base, and heel, respectively; then, the angle change of the knee joint was used as the input of the multilayer perceptron to classify the first touching position of the patient's foot, with a classification accuracy of 100% [6]. Based on the research results of this paper, it can be found that using sensor sensing technology and deep learning artificial intelligence analysis method can realize the accurate measurement and quantitative evaluation of the motor function of stroke patients, make up for the lack of traditional evaluation methods, and facilitate the development of rehabilitation evaluation in the family and community environment.

Building a virtual mechanical model or learning and forecasting existing data through neural network algorithm can better reflect the balance ability of the target population. However, the main problem at present is the lack of large sample and multidisease clinical evaluation model and its clinical feasibility needs further study.

## 2. Materials and Methods

Artificial intelligence is an important branch of computer science, which includes many application fields such as machine learning, machine vision, and intelligent search. Machine learning (ML) is the fundamental way to make computers intelligent, to put it simply. ML can be understood as enabling the computer to discover and mine deep rules from massive data and then carry out data classification and prediction, which is similar to the functional model in mathematics. The data sample is taken as the input variable, and the output is the expected result of simulation. ML can be further divided into supervised and unsupervised learning modes [7]. Unsupervised learning is to directly model the data without providing the data samples for training in advance. The ANN to be discussed is a supervised machine learning category requiring data training. See Figure 1 for the specific machine learning classification.  Figure 2 provides a visual explanation of these two concepts through the function image.

### 2.1. Evaluation of Rehabilitation

Rehabilitation assessment is a process of collecting patient history and related data; putting forward hypotheses; carrying out inspection and measurement; comparing, synthesizing, analyzing, and interpreting the results; and finally forming a conclusion and diagnosis of obstacles. Rehabilitation assessment includes all functional or ability disabilities requiring rehabilitation treatment. Through rehabilitation assessment, the location, scope, type, nature, characteristics, degree, causes, and prognosis of obstacles can be found and determined, so as to provide the basis for the formulation of clear rehabilitation goals and rehabilitation treatment plans. Correct and accurate evaluation of rehabilitation is the premise and basis for formulating correct principles, plans, and specific implementation programs of rehabilitation treatment. In addition, the effect of patients' rehabilitation treatment also needs to be reflected by the change of rehabilitation evaluation results [8–10].

The whole process of rehabilitation treatment must rely on rehabilitation assessment. Generally speaking, rehabilitation assessment mainly has the following functions: (1) seek and determine the type, degree, and cause of obstacles; (2) guide the formulation of rehabilitation treatment plan; (3) determine rehabilitation treatment programs; (4) judge the rehabilitation effect; (5) prognostic analysis; and (6) prevent the occurrence and development of obstacles. In the process of assessing various functional disorders, the commonly used rehabilitation evaluation methods include observation method, investigation method, scale method, and instrument measurement method; among them, scale method is the most commonly used evaluation method in clinical practice at present, and it is a method to use standardized scale to classify the severity of dysfunction of patients or to summarize the score.

### 2.2. Circulating Neural Network

Recurring neural network (RNN), also known as automatic association network or feedback network, is one of the most popular deep learning algorithms at present. RNN units are connected to each other in turn to form a directed cycle, and the internal state of the units makes the network show dynamic temporal behavior. They are particularly powerful in tasks where context is crucial for predicting results and are often applied to solve problems in areas such as speech recognition and natural language processing. The RNN can use its internal memory to process any input sequence. In RNN, signals propagate forward and backward by introducing a loop in the network.

The forward propagation formula of RNN is shown as follows:

(1) $$\begin{array}{c} z_{h}^{t}=\sum_{i=1}^{I}wihx_{i}^{t}+\overset{H}{\underset{h^{\prime }}{\sum }}wh^{\prime }h^{a_{h^{\prime }}{}^{t-1}}, \end{array}$$

(2) $$\begin{array}{c} a_{h}^{t}=f_{h}\left(z_{h}^{t}\right), \end{array}$$

(3) $$\begin{array}{c} y_{k}^{t}=\overset{H}{\underset{h=1}{\sum }}w_{hk}a_{h}^{t}, \end{array}$$

where lining is the input vector of neuron I in the input layer at time *t*, *a*_*h*′_^*t*−1^ is 1 moment *h*′ neurons' hidden state vectors, which are information from memory units at the previous moment, *z*_*h*_^*t*^ is the input information at time *t* and the memory unit information at the previous time obtained by weighted product and sum, after nonlinear transformation of the activation function *f*_*h*_(·). It becomes the information spit of the memory unit at the current moment. Common activation functions include Softmax, ReLU, and Tanh. *y*_*h*_^*t*^ is the output vector of K neuron in the output layer at time *t*. *w*_*ih*_, *w*_*h*′*h*_,  and *w*_*hk*_ are, respectively, the connection weights between the input layer and hidden layer, hidden layer and hidden layer, and hidden layer and output layer.

Accuracy: accurate rate can be used to represent the ability of the classifier to correctly classify samples in the whole sample set, that is, the ratio of all correctly classified samples to the total number of samples, including true positive and true negative samples, and their calculation is shown as follows:

(4) $$\begin{array}{c} \mathrm{accuracy}=\frac{\mathrm{TP}+\mathrm{TN}}{\mathrm{TP}+\mathrm{FN}+\mathrm{FP}+\mathrm{TN}}. \end{array}$$

Precision: accuracy is the percentage of samples that are predicted to be positive where the true value is also positive. It is the degree to which the predicted sample is close to the true value, and its calculation is shown in the following formula:

(5) $$\begin{array}{c} \mathrm{precision}=\frac{\mathrm{TP}}{\mathrm{TP}+\mathrm{FP}}. \end{array}$$

False positive rate (FPR) represents how many negative samples were wrongly classified as positive, calculated as follows.

(6) $$\begin{array}{c} \mathrm{FRP}=\frac{\mathrm{FP}}{\mathrm{FP}+\mathrm{TN}}. \end{array}$$

The mean square error can be understood as the Euclidean distance between the true value of the sample and the predicted value as follows:

(7) $$\begin{array}{c} \mathrm{MSE}=\frac{1}{N}\sum_{i=1}^{N}{\left(y_{i}-{\hat{y}}_{i}\right)}^{2}. \end{array}$$

Since MSE contains square operation, the value of the calculated result is very large, which is not conducive to comparative analysis. Therefore, RMSE is born, that is, the square sign of MSE is taken to make the order of magnitude of the error result consistent with the order of magnitude of the sample data as follows:

(8) $$\begin{array}{c} \mathrm{RMSE}=\sqrt{\frac{1}{N}\sum_{i=1}^{N}{\left(y_{i}-{\hat{y}}_{i}\right)}^{2}}. \end{array}$$

## 3. Results and Discussion

This data collection experiment was carried out in the Chinese Medicine Knowledge and Data Engineering Experiment of University of Electronic Science and Technology of China. The actions of the experiment were conducted under the guidance of clinical professionals, and all of them came from rehabilitation doctors with rich experience in the rehabilitation research of stroke patients and stroke rehabilitation treatment. According to the results of existing studies, at least 20 subjects (5 in each group) are required to achieve a statistical power of 0.95 in the test to detect differences in limb mobility among patients with different degrees of impairment. Therefore, a total of 36 healthy subjects (20 males, 16 females, mean age 23 ± 1.5 years) were enrolled in this study, and each participant was subjected to a Brunnstrom II–VI simulation of upper limb motor dysfunction in stroke patients.

The shoulder touch exercise was used as arm activity assessment, and the motor ability of the subjects' upper limbs was observed. Under normal circumstances, a complete movement process includes the following four steps:

1. Starting position: the subject is comfortably seated on the chair, with the torso straight, head straight, neck straight, upper limbs hanging naturally on both sides of the body (neutral position), lower limbs naturally relaxed, and knees bent 90°
2. Lift the hemiplegic arm on the sagittal plane to horizontal height (shoulder flexion 90°)
3. Bend the elbow and touch the opposite shoulder with the palm of your hand (elbow flexion and forearm pronation)
4. The upper limbs naturally return to the starting position (shoulder extension, elbow extension, and forearm pronation); therefore, the number of data samples in each period is equal to 36; a total of 180 samples were identified

In the simulation data collection stage, Figure 3 shows the sample triaxial acceleration data collected by two IMU of forearm and upper arm during the Brunnstrom II–VI simulation of movement disorders of the same subject. The solid line is the triaxial acceleration data collected by the IMU at the forearm position, while the dashed line is the triaxial acceleration data of the IMU at the forearm position. As can be seen from Figure 3, due to the different severity, the patient's arm presents different distribution rules in the process of performing the same activity. Stage II patients have higher severity, and the upper limb joints cannot realize a full range of activities.

From Figure 4, we first observe that the deep learning model based on the cyclic neural network has better performance than the linear model in all indicators. As for the logistic regression model, its average accuracy in 5 categories was 27.80%, with an average AUROC of 0.53 and AUPRC of 0.35, which was the worst performance among all models. This is consistent with previous research results that compared the neural network with linear model of time series data. Deep learning method has more and more complex parameters than the traditional learning method and can extract richer and more accurate features by itself.

In order to further prove the performance effect of the proposed method, we analyze the confusion matrix on the test set of all the methods.  Table 1 denotes the confusion matrix of TARM and LR classification results on the test set. The TARM was consistent in classifying data for each Brunnstrom stage, and patients with stage III and IV injuries, depending on the location of the injury. The upper limb movements are more complex than those of other stage patients, leading to unstable data classification of these stages in the LR model.

## 4. Conclusions

Evaluation of rehabilitation is an important link in the process of rehabilitation treatment, which is the basis for the establishment of rehabilitation program and the evaluation of rehabilitation effect. In view of the upper limb motor dysfunction that often occurs after stroke, based on the objectivity and performance defects of the existing clinical rehabilitation evaluation methods and automatic evaluation research, deep learning technology was first applied to the automatic evaluation research of stroke rehabilitation. Firstly, the commonly used clinical scales are analyzed, and the motion measurement system is designed according to the evaluation project content and scoring requirements. Then, different depth learning algorithm models are output according to the data characteristics and expected output. Finally, this automatic evaluation research is compared with relevant depth learning algorithms to verify that the proposed method is a better method for realizing the automatic evaluation task of upper limb motor function. Experiments showed that the trained ANN had the same score as human for most of the data (82.2%, Cohen's kappa = 0.743). There was a strong correlation between ANN and improved Ashworth scores as assessed by human raters (*r* = 0.825, *p* < 0.01). These characteristics of ANN can help it to learn a large number of clinical data and then generate a stable clinical evaluation model, improve the accuracy and efficiency of rehabilitation evaluation, reduce the work intensity of rehabilitation physicians and therapists, and alleviate the current shortage of rehabilitation resources. Using measurement methods, although the degree of interference is low, it is easy to produce measurement error, affect the quality of the data, missing values, and other problems. In terms of data analysis, the data collected by neural network lack missing processing.

## Figures and Tables

**Figure 1:** Machine learning classification.The ANN to be discussed is a supervised machine learning category requiring data training.

**Figure 2:** Fitting function simulation provides a visual explanation of these two concepts through the function image.

**Figure 3:** Sample IMU acceleration data of subjects at different stages. Due to the different severity, the patient's arm presents different distribution rules in the process of performing the same activity.

**Figure 4:** Sample data of subject's forearm IMU sensor. As for the logistic regression model, its average accuracy in 5 categories was 27.80%, with an average AUROC of 0.53 and AUPRC of 0.35.

**Table 1:** Brunnstrom staging confusion matrix (TARM).

		Ground truth					Classified sum
Prediction	Stage II	Stage II	Stage III	Stage IV	Stage V	Stage VI	
	Stage III	7	0	0	0	0	7
	Stage IV	0	9	0	0	0	9
	Stage V	0	3	0	0	0	9
	Stage VI	0	0	0	0	6	6
No. of samples		7	9	9	6	5	5
Accuracy		100%	100%	100%	100%	100%	

## Data Availability

The data used to support the findings of this study are available from the corresponding author upon request.

## References

[1] Min K., Beom J., Kim B. R. (2021). Clinical practice guideline for postoperative rehabilitation in older patients with hip fractures. *Annals of Rehabilitation Medicine*.

[2] Suwarno S. (2019). Performance evaluation of artificial neural network classifiers for predicting cesarean sections. *International Journal of Scientific & Technology Research*.

[3] Vukicevic A. M., Jovicic G. R., Jovicic M. N., Milicevic V. L., Filipovic N. D. (2018). Assessment of cortical bone fracture resistance curves by fusing artificial neural networks and linear regression. *Computer Methods in Biomechanics and Biomedical Engineering*.

[4] Papathanasiou J. V., Carraro U. (2018). Postoperative rehabilitation of elderly patients. *Practical Issues in Geriatrics*.

[5] Pryor M., Carrion R., Wang R., Henry G. (2016). 066 prospective evaluation of postoperative penile rehabilitation: penile morphology and patient satisfaction 2 Years following coloplast titan inflatable penile prosthesis. *The Journal of Sexual Medicine*.

[6] Wilkinson B. G., Donnenwerth J. J., Peterson A. R. (2019). Use of blood flow restriction training for postoperative rehabilitation. *Current Sports Medicine Reports*.

[7] Morey A. F., Allen F. (2016). Re: prospective evaluation of postoperative penile rehabilitation: penile length/girth maintenance 1 year following coloplast titan inflatable penile prosthesis. *The Journal of Urology*.

[8] Dusenberry M. W., Brown C. K., Brewer K. L. (2017). Artificial neural networks: predicting head ct findings in elderly patients presenting with minor head injury after a fall. *The American Journal of Emergency Medicine*.

[9] Ilves O., HKkinen A., Dekker J. (2017). Quality of life and disability: can they be improved by active postoperative rehabilitation after spinal fusion surgery in patients with spondylolisthesis? a randomised controlled trial with 12-month follow-up. *European Spine Journal*.

[10] Ilves O., Hakkinen A., Dekker J. (2017). Quality of life and disability: can they be improved by active postoperative rehabilitation after spinal fusion surgery in patients with spondylolisthesis? A randomised controlled trial with 12-month follow-up. *European Spine Journal*.

